# Serum Levels of S100A11 and MMP-9 in Patients with Epithelial Ovarian Cancer and Their Clinical Significance

**DOI:** 10.1155/2021/7341247

**Published:** 2021-03-03

**Authors:** Wenjing Li, Zhumei Cui, Yan Kong, Xiangyu Liu, Xiangyu Wang

**Affiliations:** ^1^Department of Gynecology, The Affiliated Hospital of Qingdao University, Qingdao University, Qingdao, China; ^2^Department of Gynecology, The Affiliated Hospital of Qingdao University, Qingdao, Shandong Province, China

## Abstract

**Objective:**

To investigate the serum levels of calgizzarin (S100A11) and matrix metalloproteinase-9 (MMP9) in patients with epithelial ovarian cancer (EOC) and determine their clinical significance.

**Methods:**

Serum levels of S100A11 and MMP9 were detected in patients with EOC, patients with benign ovarian tumor, and healthy women. The correlation between the two markers and clinicopathological characteristics of ovarian cancer was analysed.

**Results:**

The serum levels of S100A11 and MMP-9 in patients with EOC were higher than those in patients with benign ovarian tumor and in healthy women, and the expression levels of S100A11 and MMP-9 were positively correlated. S100A11 and MMP-9 were correlated with tumor staging, postoperative residual foci, ascites volume, serum CA125 level, chemotherapy response, and lymph node metastasis, while S100A11 and MMP-9 were not associated with the bilevel classification, histological type, age, and degree of differentiation.

**Conclusion:**

S100A11 and MMP-9 were both highly expressed in the serum of patients with EOC and were associated with cancer development, invasion, and metastasis. Therefore, they can be used as an important reference maker in the diagnosis and treatment of ovarian cancer.

## 1. Introduction

EOC is the most common type of ovarian cancer; it has a high degree of malignancy and an insidious onset, and the long-term survival rate remains at 20-30% [1]. Most patients are diagnosed at the late stage of cancer and miss the optimal timing for surgery. Therefore, the search for definitive early diagnostic indicators is of great significance for the diagnosis, treatment, and prognosis of patients with ovarian cancer. As in the case of other malignant tumors, tumor invasion and metastasis are important factors affecting the prognosis of patients with EOC. The occurrence and development of EOC is a multifactorial, multistage, complex process that is affected by many factors [2]. The origin and pathogenesis of ovarian cancer have not yet been elucidated. Further understanding of the molecular mechanisms of ovarian cancer may lead to the more effective development of treatment strategies.

S100A11 is a multigene family of EF-hand calcium-binding proteins. S100A11 is an important member of the S100 protein family. It is mainly involved in the regulation of cell-signaling pathways but also plays a role in cell growth, proliferation, differentiation, and apoptosis and is closely associated with tumors. It has been reported that high expression of the S100A11 gene in some tumors can upregulate the expression of MMP-9, thus promoting tumor invasion [3]. MMP-9 is a member of the matrix metalloproteinase family. As an important proteolytic enzyme, MMP-9 is involved in tumor invasion and metastasis. Through the degradation of the extracellular matrix, it accelerates the infiltration of cancerous cells into surrounding tissues [4]. Currently, there are few studies on the expression of S100A11 and MMP9 in EOC, and the clinical correlation between S100A11 and MMP9 is also not clear [5]. In this study, enzyme-linked immunosorbent assay (ELISA) was used to detect the levels of serum S100A11 and MMP9 in patients with EOC, patients with benign ovarian tumor, and healthy women to explore the correlation between the two potential markers and their relationship with EOC invasion and metastasis.

## 2. Materials and Methods

### 2.1. Patient Samples

A total of 111 patients with EOC who were diagnosed and treated at the Department of Obstetrics and Gynaecology at the Affiliated Hospital of Qingdao University, China, between November 2010 and January 2020 were included in this study. Thirty patients with benign ovarian tumors and 25 healthy women who underwent physical examinations during the same period were included as controls. The subjects were between 34 and 74 years old, with a median age of 51 years. The pathological diagnosis of all EOC patients was confirmed by two experienced pathologists. Surgical staging was carried out according to the staging criteria of the International Federation of Gynaecology and Obstetrics (FIGO) [6]. None of the subjects had a history of chemotherapy, radiotherapy, or immunotherapy before specimen collection. The samples were classified based on clinicopathological parameters, including age at initial diagnosis, FIGO stage, histological subtype, histological grade, ascites volume, serum CA125 level, postoperative residual tumor mass size, and chemotherapy response. Aside from one stage I G1 patient, the EOC patients received cytoreductive surgery and paclitaxel plus platinum-based chemotherapy. Patients were grouped according to the assessment of their chemotherapy response [7] and the dualistic theory of ovarian cancer [8]. This study was approved by the Ethics Committee of the Affiliated Hospital of Qingdao University (approval number: QYFYWZLL 26079). All patients or their relatives signed written informed consent.

### 2.2. Method

Early in the morning before surgery, 8 mL of fasting peripheral blood was collected from the subjects and centrifuged at 2000 g for 10 min. The separated serum was stored in a -80°C freezer for subsequent measurement. The levels of S100A11 and MMP9 in peripheral blood were measured using the MMP-9 ELISA kit from R&D (USA) and the S100A11 ELISA kit from BioVendor.

### 2.3. Statistical Analysis

SPSS 25.0 was used for data analysis. The data obtained in this study were measurement data. The Shapiro-Wilk test was used to assess the distribution of normality. Since the data were not normally distributed, median (P25-P75) was used for the data description. The Kruskal-Wallis or Mann–Whitney *U* test was used to compare and analyse different groups. The Bonferroni correction method was used for comparisons between groups. Spearman's rank correlation analysis was used for correlation analysis. *P* < 0.05 was considered statistically significant.

## 3. Results

### 3.1. Expression Levels of S100A11 and MMP-9 in the Serum of Each Group

The serum levels of S100A11 and MMP-9 in the malignant group were significantly higher than those in the benign group and the healthy control group (*P* < 0.05). The levels of S100A11 and MMP-9 in the peripheral blood of the benign group were significantly higher than the levels in the healthy control group (*P* < 0.05) (Table 1).

### 3.2. Correlation between S100A11, MMP-9, and Other Clinicopathological Features of EOC Patients

High serum S100A11 levels in EOC patients were closely related to tumor pathological stage, postoperative residual foci, ascites volume, serum CA125 level, platinum-based chemotherapy response, and lymph node metastasis (*P* < 0.05). Similarly, high serum MMP-9 levels were also closely related to the aforementioned six factors (*P* < 0.05). Conversely, S100A11 and MMP-9 expression in the peripheral blood of EOC patients was not associated with the bilevel classification or the classification of EOCs, histological type, age, or degree of differentiation (*P* > 0.05). The serum levels of S100A11 and MMP-9 in patients with late-stage (stage III-IV) EOC were higher than those of patients in the early stage (stage I-II); the expression levels of S100A11 and MMP-9 in the serum of patients with lymph node metastasis were higher than the serum levels of patients without metastasis; the expression level of S100A11 and MMP-9 in the serum was high in patients with a large volume of ascites or large residual tumor foci. The expression levels of S100A11 and MMP-9 were higher in chemotherapy-insensitive patients than in chemotherapy-sensitive patients, and all differences were statistically significant (*P* < 0.05) (Table 2).

### 3.3. Correlation between Serum S100A11 and MMP-9 in EOC Patients

Spearman's rank correlation analysis showed a significant positive correlation between serum S100A11 and MMP9 in EOC patients (rs = 0.405, *P* < 0.05).

## 4. Discussion

Due to the lack of specific clinical manifestations and effective screening methods, ovarian cancer is difficult to detect and diagnose at an early stage. Most patients have an excellent response to platinum-based drugs at the initial treatment, but almost all patients with advanced ovarian cancer will relapse and will progress to platinum resistance after multiple relapses [9]. Targeted drugs have been written into ovarian cancer treatment guidelines [10] and are expected to make ovarian cancer a controllable chronic disease, though it still cannot be cured. The mortality rate of ovarian cancer remains the highest among gynaecologic tumors. A common challenge facing various treatment regimens for ovarian cancer is the lack of effective biomarkers.

S100A11, also known as S100C or calgizzarin, is an important member of the S100 family [11]. A number of cancers have been reported to involve overexpression of S100A11, including thyroid cancer [12], colon cancer [13], pancreatic cancer [14], and breast cancer [15]. The study of Shankar et al. [16] showed that the reduction or deletion of S100A11 expression could lead to an interaction between cells and E-cadherin protein expression, thereby reducing tumor migration and invasion. S100A11 also has high expression in ovarian cancer cells. Knocking out the S100A11 gene could inhibit the growth, invasion, and migration of ovarian cancer cells [17].

The degradation of the extracellular matrix is a crucial step in the invasion and metastasis of malignant tumors. MMP-9 has the largest molecular weight among the MMPs, and it can degrade almost all the extracellular matrix components, causing weakening of the adhesion between tumor cells and damaging barriers that prevent cancer cell invasion and metastasis, thus providing sufficient space for cancer cells to spread and metastasize to distant regions and promoting tumor growth, infiltration, and metastasis [18]. Wood et al. [19] confirmed that MMP-9 is involved in the tumorigenesis, invasion, and metastasis processes of a variety of tumors. Therefore, inhibition of S100A11 and MMP-9 expression may further inhibit tumor invasion and metastasis, providing a promising direction in the diagnosis and treatment of ovarian cancer patients.

The experimental results showed that high serum S100A11 and MMP-9 expression was associated with high CA125 and a large volume of ascites. CA125 is an important biomarker of EOC [20], and ascites is also considered an important indicator in the diagnosis, treatment, and follow-up of EOC [21]. These results preliminarily confirmed that S100A11 and MMP-9 were associated with CA125 and ascites, suggesting that S100A11 and MMP-9 were closely related to the progression of EOC. The monitoring of S100A11 and MMP-9 levels is helpful for EOC diagnosis, efficacy evaluation, and prognosis evaluation.

Chemoresistance is considered to be the main reason for treatment failure in EOC patients and is an important indicator for determining the prognosis of EOC in clinical practice [22]. Studies have shown that in ovarian cancer cells with high MMP-9 expression, the combined use of MMP9/MMP2 inhibitors and cisplatin could significantly enhance cytotoxicity, confirming that MMP9 is a potential therapeutic target for drug-resistant ovarian cancer [23]. S100A11 has also been confirmed to be associated with drug resistance in tumors. Zagresjzzaya et al. [24] found that low S100A11 expression promoted reactive oxygen species- (ROS-) dependent cell apoptosis through the activation of phospholipase A2 (PLA2), thereby enhancing the sensitivity of lung cancer cells to cisplatin, 5-fluorouracil, and oxaliplatin. In this study, all patients except the one with FIGO stage IG1 cancer received paclitaxel plus platinum-based adjuvant chemotherapy after cytoreductive surgery. The results showed that elevated levels of S100A11 and MMP-9 were associated with chemoresistance. This finding is consistent with previous experimental results, suggesting that S100A11 and MMP9 are potential therapeutic targets for drug-resistant ovarian cancer. Therefore, the joint analysis of S100A11 and MMP-9 is very important in the study of drug-resistance mechanisms in ovarian cancer.

## 5. Conclusions

The results of this study showed that S100A11 and MMP-9 expression in the peripheral blood of EOC patients was significantly higher than that in patients with benign ovarian cancer and healthy controls. S100A11 and MMP-9 levels were low in the control group but were elevated in early-stage tumors and reached the highest level in advanced tumors. Statistical analysis showed that high expression of S100A11 and MMP-9 was positively correlated with the FIGO stage and lymph node metastasis of EOCs, suggesting that S100A11 and MMP-9 play important roles in the occurrence and development of EOCs and are closely associated with prognosis, thus suggesting a new therapeutic target for ovarian cancer. However, whether S100A11 and MMP-9 can be used as a biological indicator for early screening and the long-term postoperative follow-up of malignant changes in EOC still deserves further exploration. Our next step is to investigate the biological roles and mechanisms of S100A11 and MMP-9 in EOCs to assist in clinical diagnosis and treatment and to improve the prognosis of patients.

## Figures and Tables

**Table 1:** Expression levels of S100A11 and MMP-9 in the serum of each group.

Group	No. of patients	S100A11 (ng/mL)	MMP-9 (ng/mL)
Healthy control group	25	5.02(1.54-7.19)	89.63(7.28-209.47)
Benign group	30	8.41 (5.12-14.85)	122.95 (54.99-256.26)
Malignant group	111	14.54 (4.46-38.86)	189.71 (35.21-688.99)

The Kruskal-Wallis test was used to compare different groups: the serum levels of S100A11 in malignant group compared with control group and benign group, *P* < 0.05; the serum levels of MMP-9 in malignant group compared with control group and benign group, *P* < 0.05.

**Table 2:** The relationship between the serum levels of S100A11 and MMP-9 and clinicopathological characteristics in patients with EOC.

Clinical variable	No. of patients	S100A11 (ng/mL) Median (range)	*P* value^a^	MMP-9(ng/mL) Median (range)	*P* value^a^
All cases	111				
Age at diagnosis(years)			0.201		0.136
<51	55	11.01 (4.46-32.74)		165.53 (35.21-688.99)	
≥51	56	15.60 (5.60-38.86)		199.61 (59.01-475.02)	
Histological type			0.32		0.678
Serous	80	13.41 (4.46-32.22)		180.51 (35.21-475.02)	
Mucinous	10	12.58 (7.60-32.75)		195.80 (63.42-688.99)	
Endometrioid	13	10.75 (6.38-38.86)		151.90 (47.22-422.59)	
Clear cell tumor	8	12.32 (8.13-29.86)		153.26 (55.59-248.06)	
Tumor grade			0.93		0.978
G1	8	13.02 (8.03-22.62)		182.96 (63.42-441.95)	
G2	23	11.71 (6.38-32.22)		156.85 (47.22-422.59)	
G3	80	13.02 (4.46-38.86)		181.38 (35.21-688.99)	
Lymph node metastasis			0.01		0.007
Negative	60	12.58 (4.46-32.75)		154.03 (35.21-688.99)	
Positive	51	14.24 (5.60-38.86)		204.23 (63.47-475.02)	
FIGO stage			<0.001		<0.001
I, II	30	10.00 (6.38-29.86)		139.94 (43.82-246.16)	
III, IV	81	14.15 (4.46-38.86)		199.65 (35.21-688.99)	
Serum CA125 level (U/mL)			0.04		0.002
<35	26	12.32 (4.46-31.26)		154.44 (35.21-441.95)	
≥35	85	14.29 (6.20-38.86)		199.59 (43.82-688.99)	
Chemotherapy resistance^b^			0.01		<0.001
Present	31	12.32 (4.46-31.26)		154.44 (35.21-441.95)	
Absent	79	14.29 (6.20-38.86)		199.59 (43.82-688.99)	
Ascites (mL)			0.01		0.045
<500	51	12.32 (4.46-31.26)		154.44 (35.21-441.95)	
≥500	60	14.29 (6.20-38.86)		199.59 (43.82-688.99)	
Two-tier system			0.52		0.29
I type	45	12.76 (6.38-38.86)		156.85 (47.22-441.95)	
II type	66	13.19 (4.46-32.75)		183.62 (35.21-688.99)	
Residual tumor size (cm)			0.03		0.002
<2	86	12.76 (4.46-38.86)		167.70 (35.21-688.99)	
≥2	25	15.81 (5.60-31.17)		244.50 (83.18-344.22)	

^a^The Mann–Whitney *U* and Kruskal-Wallis nonparametric tests were used to compare different groups. ^b^One patient with stage I and Grade I did not undergo chemotherapy.

## Data Availability

All the data can be available by asking from the corresponding author.
